RETRACTED

# Granulocyte colony stimulating factor versus human chorionic gonadotropin for recurrent implantation failure in intra cytoplasmic sperm injection: a randomized clinical trial

**DOI:** 10.1186/s12884-022-05098-9

**Published:** 2022-11-29

**Authors:** Mohamed Sobhy Bakry, Elsayed Eldesouky, Moatazza Mahdy Alghazaly, Elsayed farag, Eslam Elsayed Kamal Sultan, Hossam Elazzazy, Attia Mohamed, Soliman Mohamed Said Ali, Assem Anwar, Asmaa Ahmed Elrashedy, Mohamed Abdelmonem, Mohamed Abd-ElGawad, Almandouh H. Bosilah

**Affiliations:** 1 Department of Obstetrics and Gynecology, Faculty of Medicine, Fayoum University, Fayoum, Egypt; 2 Department of Obstetrics and Gynecology, Faculty of Medicine, Alazhar University, Cairo, Egypt; 3 Department of Obstetrics and Gynecology, Faculty of Medicine Girls, Alazhar University, Cairo, Egypt; 4 Department of Obstetrics and Gynecology, Faculty of Medicine, Alazhar University, Domiata, Egypt; 5 Faculty of Medicine, Kafr El-Shaikh University, Kafr El-Shaikh, Egypt; 6 Faculty of Medicine, Fayoum University, Fayoum, Egypt; 7 Department of Obstetrics and Gynecology, Faculty of Medicine, Domiata University, Domiata, Egypt

**Keywords:** RIF, G-CSF, HCG, ICSI, IVF

## Abstract

**Background:**

Repeated implantation failure (RIF) is defined as the case whereby the transferred embryos fail to implant after several attempts of In vitro fertilization (IVF) which causes a profound impact on the quality of life and financial burden. Some clinical studies have confirmed that Granulocyte colony-stimulating factor (G-CSF) and human chorionic gonadotropin (HCG) can improve pregnancy outcomes and implantation rates. Hence, our study aims to compare the efficacy of G-CSF and HCG on pregnancy outcomes in RIF women who undergo intra-cytoplasmic sperm injection (ICSI).

**Methods:**

This randomized, single-blinded study was conducted et al.-Azhar University Hospitals, Cairo, Egypt, between 10^th^ October 2020 and 20^th^ December 2020. The study included 100 women aged 20–43 years old undergoing ICSI cycles, with a history of RIF. Patients were divided randomly into two groups: group (1): included 50 patients injected with 500 IU of intrauterine HCG on embryo transfer day, and group (2): Included 50 patients injected with G-CSF on the embryo transfer day.

**Results:**

In 100 RIF women, we found a significant improvement in pregnancy outcomes favoring G-CSF over HCG including implantation rate, chemical pregnancy, and clinical pregnancy (*P* < 0.0001, *P* = 0.0003, and *P* = 0.0006, respectively).

**Conclusion:**

For the first time, we demonstrated a significant improvement in pregnancy outcomes favoring G-CSF over HCG in terms of implantation rate, chemical pregnancy, and clinical pregnancy.

RETRACTED

**Trial registration:**

The study was registered on Pan African Clinical Trials Registry with the following number: PACTR202010482774275 and was approved on 2^nd^ October 2020.

## Background

Recurrent implantation failure (RIF) affects patients who undergo assisted reproductive technology (ART). RIF is defined as clinical pregnancy failure after implanting four high-quality embryos in women aged below 40 years old and after undergoing three fresh or frozen cycles of in vitro fertilization (IVF) resulting in a significant reduction in life quality and economic burden [1, 2].

The exact incidence of RIF is unknown and it is affected by many factors such as women's ages; increased weight; anatomical deformities; lifestyle factors including smoking, pollutants exposure, and stress; genetic background; thrombophilia; ART-associated factors; and autoimmune diseases [3].

Over the last few decades, developments in ART resulted in significant increases in IVF/intracytoplasmic sperm injection (ICSI) pregnancy rates [4]. As vitrification technologies and pre-implantation genetic diagnostics were improved, researchers better grasped one of the two crucial elements in the RIF process: the embryo and the endometrium which corrected a mistaken idea of the success of pregnancy required a healthy embryo only irrespective of endometrium condition [3, 5].

The receptive healthy endometrium allows changing of endometrial cells into decidua cells, blastocyst invasion, and fast placental expansion [6]. Other factors increase implantation rates including Immune cells, growth factors, cytokines, and hormonal changes [7].

Granulocyte colony-stimulating factor (G-CSF) is produced in the maternofetal interaction during embryo implantation in early pregnancy, suggesting that it may be involved in decidua and placental functionality [8]. G-CSF receptor expression increases throughout pre-ovulatory follicle maturation, in human endometrium, and in luteinized granulosa cells [9]. It activates intracellular pathways involved in the proliferation, differentiation, and stimulation of neutrophilic granulocyte lineage hematopoietic cells [10]. It also affects cytokine production from type two T helper cells, activates T regulatory cells, affects cytotoxicity of the uterine natural killer cells, and increases endometrial angiogenesis which plays an essential part in early embryo-uterine endometrium cross-talk [9].

The management of RIF is currently being investigated as recommended by treatments including G-CSF in addition to Human Chorionic Gonadotropin (HCG) which is a glycoprotein hormone released by placental syncytiotrophoblasts and keeps the production of progesterone by corpus luteum [11, 12]. Two-cell stage embryos already secrete the HCG-subunits, and their concentrations rise to high levels in blastocysts [13]. As a result, HCG triggers the interaction between embryo and endometrium before embryo entrance as a day five or six blastocysts into the uterine cavity. Also, it modulates women's immune reactions during implantation [14]. Patients with RIF, on the other hand, have significantly lower percentages of Regulatory T cells (Tregs) [15]. Tregs are required for maternal–fetal tolerance to be maintained. The HCG hormones boost Tregs in the periphery during pregnancy and draw them to maternal–fetal contact [16]. Hence, our study aimed to compare the efficacy of G-CSF and HCG in RIF women who have undergone ICSI on pregnancy outcomes such as implication rate, chemical pregnancy, and clinical pregnancy.

RETRACTED

## Methods

### Study design and study population

This randomized, single-blinded study was performed et Al-Azhar University Hospitals in Cairo, Al-Azhar University Hospitals of Assiut, Al-Azhar University Hospitals of Damietta, Dar Eltib Fertility Center, Ahmed Oraby Fertility Center, and Wald we Bent Fertility Center between 10^th^ October 2020 and 20^th^ December 2020. The study was approved by ethics committee of the Quality Education Assurance Unit et al. Azhar Faculty of Medicine and all patients gave informed consent before enrollment. The study's protocol was registered on Pan African Clinical Trials Registry with the following number: PACTR202010482774275 and was approved on 02/10/2020. The inclusion criteria were women aged 20–43 years with a history of RIF who undergoing ICSI cycles. RIF was determined by clinical pregnancy failure after three cycles of IVF. Women with associated medical disorders were excluded as diabetes, hypertension, heart diseases, and thyroid disorders. Included patients were blinded to their group. They were divided by simple randomization generated by a computer program and were allocated by sealed opaque envelops into two parallel groups: group (1): 50 patients injected with 500 IU of intrauterine HCG on embryo transfer day, and group (2): 50 patients injected with G-CSF on embryo transfer day. Only the participants and outcome assessors were blinded while the caregivers were not blinded.

### Sample size calculation

We used MedCalc® 12.3.0.0 "Ostend, Belgium" software to estimate the required included sample. The sample size was adjusted by confidence interval = 95%, margin of error = 5%, and study's power = 80%. The estimated pregnancy rate was 18 (56.2%) for G-CSF group and 8 (40%) for control group as presented in Arefi et al. with *P*-value = 0.09 [17]. Therefore, according to these values, the least number of included patients that could produce a difference between the two groups was 100 patients with 50 patients for the HCG group and 50 patients for the G-CSF group.

RETRACTED

### Treatment protocol

On the second day of the cycle, all patients had a transvaginal ultrasound examination to examine antral follicle count (AFC). Also, we measured the levels of the following hormones: Follicle Stimulating Hormone (FSH), Prolactin, Luteinizing Hormone (LH), Thyroid Stimulating hormone (TSH), Estradiol (E2), and Anti-Müllerian Hormone (AMH). Then, they started the gonadotropin-releasing hormone (GnRH) agonist protocol which was started from the mid-luteal phase and was continued until HCG triggering day by subcutaneous administration of 0.1 mg Decapeptyl (Ferring Pharmaceuticals, Germany) per day. After down regulation of pituitary gland which was determined by decreasing E2 serum concentration below 50 pg/ml, the ovarian stimulation was started on the second day of menstrual bleeding with intramuscular injection (IM) of (75 – 300) IU Human Menopausal Gonadotropins (HMG) (Merional, IBSA, Switzerland) and was continued till HCG administration day. The doses of both HMG and Decapeptyl were adjusted according to the characteristics of the patients such as age and body mass index or clinical progress by AFC. By the sixth cycle day, transvaginal ultrasound was performed every three days to evaluate the ovarian progress then the imitating HMG dose was estimated according to the concentration of E2 in the patients' sera.

All patients were administered 10,000 IU of HCG (Choriomon, IBSA Pharmaceutical, Switzerland) when the mean diameter of follicles became more than (18 – 24) mm. We extracted the oocytes after 36 h of injection of HCG guided by transvaginal ultrasound.

On the day of embryo transfer, the first group was administered by intrauterine infusion of HCG by Wallace embryo replacement soft catheter (Smiths Medical International Ltd., UK). The HCG was prepared by adding one 5000 IU vial to 10 ccs isotonic saline, therefore every one cm contained 500 IU HCG. The second group was administered 300 mcg/ 1.0 G-CSF (Geneleukin) by using the same technique as the first group as one cc from it was diluted by adding dextrose 5% by ratio = 1:2, therefore every one cc contained 100 mcg. In the end, pelvic ultrasound was conducted to exclude any internal bleeding.

After performing fertilization procedures, we transferred one to three grade A embryos on the fifth day of fertilization. Then, we started administration of 400 mg of cyclogest vaginal suppositories (Actavis pharmaceutical, UK) at the oocyte retrieval day for luteal phase support till the performance of the serum pregnancy test (β-HCG) which was conducted after 14 days from embryo transfer. Figure 1 shows the details of the treatment procedure.

RETRACTED

### Outcomes

The primary outcome was clinical pregnancy rate which was proven by transvaginal ultrasound screening of embryos, fetal cardiac beatings, or gestational sacs at the 8th week and 14 days following the embryo transfer. The secondary outcomes were chemical pregnancy (proven with positive values of HCG according to laboratory standardized values) and implantation rate (proven with gestational sacs number that was detected by ultrasound at six weeks after pregnancy divided by transferred embryos number).

### Statistical analysis

We used SPSS versions 22, IBM, USA to perform the analysis after the recording of data. Qualitative variables were presented by number (n) and percentage (%). Quantitative variables with parametric distribution were presented as mean ± standard deviation (SD). We used the student t-test in comparative analysis of continuous variables and the Chi-square test in comparative analysis of categorical variables. The outcomes were considered to be significant when *P*-value was < 0.05.

## Results

We recruited the patients from 10^th^ October 2020, and 20^th^ December 2020 and one hundred patients with RIF were eligible and included: 50 patients (50%) in the G-CSF group and 50 patients (50%) in the HCG group (Fig. 2). All patients were followed up for two months. The demographic characteristics and pre-cycle identifiers of these individuals and their spouses are shown in Table 1. No differences were observed between groups regarding patient age, husband age, body mass index, type, causes, duration of infertility, the number of previous ICSI trials, AFC, baseline endometrial thickness, and endometrial thickness at the day before HCG triggering. Also, the hormonal levels showed no significant difference between the studied groups regarding FSH (*P* = 0.107), LH (*P* = 0.347), E2 (*P* = 0.783), AMH (*P* = 0.769), prolactin (*P* = 0.325) and TSH levels (*P* = 0.653) (Table 1).

**Fig. 1:** Treatment procedure details

**Fig. 2:** CONSORT flow diagram of the included patients

**Table 1:** Comparison between Granulocyte Colony Stimulating Factor (GCSF) and Human Chorionic Gonadotropin (HCG) according to baseline characteristics, ultra-sonographic data, and laboratory data

Parameters	GCSF group (*n* = 50)	HCG group (*n* = 50)	t/X2	*P*-value
**Age (years)**			1.120	0.135
Mean ± SD	34.76 ± 4.88	32.94 ± 3.91		
Range	23–43	24–39		
**Weight (kg)**			0.013	0.858
Mean ± SD	83.84 ± 15.11	83.46 ± 16.19		
Range	54–111	52–122		
**Height (m)**			1.616	0.189
Mean ± SD	1.72 ± 0.07	1.69 ± 0.08		
Range	1.62–1.87	1.4–1.85		
**Husband Age**			1.527	0.126
Mean ± SD	40.50 ± 7.52	37.66 ± 5.45		
Range	30–59	27–50		
**Body Mass Index**			0.348	0.943
Mean ± SD	29.68 ± 6.09	29.25 ± 6.38		
Range				
**Duration of Infertility**			0.627	0.388
Mean ± SD	7.08 ± 2.65	7.60 ± 3.51		
Range	3–12	3.5–18		
**Type of Infertility**			0.051#	0.822
Primary	36 (72%)	37 (74%)		
Secondary	14 (28%)	13 (26%)		
**Cause of infertility**			0.187#	0.769
Male	10 (20%)	13 (26%)		
Ovarian	2 (4%)	4 (8%)		
Polycystic ovary	11 (22%)	8 (16%)		
Tubal	8 (16%)	6 (12%)		
Unexplained	19 (38%)	19 (38%)		
**Previous ICSI**			0.528	0.426
Mean ± SD	3.38 ± 0.53	3.48 ± 0.76		
Range	3–5	2–6		
**AFC**			1.205	0.124
Mean ± SD	9.62 ± 2.47	10.68 ± 4.25		
Range	5–14	4–20		
**Baseline Endometrial** Thickness			0.134	0.667
Mean ± SD	4.24 ± 0.78	4.17 ± 0.83		
Range	2.8–5.2	1–5		
**Endometrial Thickness before HCG** **triggering**			0.310	0.533
Mean ± SD	10.18 ± 1.43	9.97 ± 2.07		
Range	7.3–13	2.7–16		
**FSH**			1.300	0.107
Mean ± SD	7.37 ± 1.81	8.32 ± 1.93		
Range	2.7–10	5.5–12		
**LH**			0.752	0.347
Mean ± SD	0.88 ± 0.66	1.00 ± 0.62		
Range	0.1–2.8	0.1–2.8		
**E2**			0.045	0.783
Mean ± SD	28.40 ± 10.050.053	27.98 ± 8.74		
Range	18–57	16–52		
**AMH**			0.053	0.769
Mean ± SD	2.08 ± 1.03	2.02 ± 1.19		
Range	0.8–4.2	0.1–4.9		
**Prolactin**			0.831	0.325
Mean ± SD	20.48 ± 6.58	19.26 ± 6.18		
Range	10–32	7–31		
**TSH**			0.148	0.653
Mean ± SD	2.65 ± 0.88	2.57 ± 0.96		
Range	0.1–4.9	0.6–4.8		

Comparison between Granulocyte Colony Stimulating Factor (GCSF) and Human Chorionic Gonadotropin (HCG) according to baseline characteristics, ultra-sonographic data, and laboratory data

^#^ or X2 refers to chi-square test result. t refers to student t-test

*ICSI* Intracytoplasmic Sperm Injection, *FSH* Follicle Stimulating Hormone, *LH* Luteinizing Hormone, *E2* Estradiol, *AMH* Anti-Müllerian Hormone, *TSH* Thyroid Stimulating Hormone, *SD* Standard Deviation, *AFC* Antral Follicle Transfer

The characteristics of the ICSI parameters of our study are given in Table 2, with a comparison of the G-CSF and HCG groups. No statistically significant difference was identified between the two groups regarding Oocyte Retrieval Day (*P* = 0.658), Gonadotropins Dose (*P* = 0.711), and the number of embryos transferred (*P* = 0.365) (Table 2).

RETRACTED

**Table 2:** Comparison between Granulocyte Colony Stimulating Factor (GCSF) and Human Chorionic Gonadotropin (HCG) according to ICSI parameters

Parameters	GCSF group (*n* = 50)	HCG group (*n* = 50)	t/X2	*P*-value
HCG injection day (day)*			1.195	0.117
Mean ± SD	10.84 ± 1.27	10.36 ± 0.75		
Range	9–13	9–12		
**Oocyte Retrieval (hours)†**			0.890	0.309
Mean ± SD	35.90 ± 1.02	35.74 ± 0.53		
Range	33–39	34–36		
**Gonadotropins Dose (IU)**			0.094	0.711
Mean ± SD	32.12 ± 5.05	31.86 ± 2.70		
Range	20–42	27–39		
**Retrieved oocytes**			1.431	0.202
Mean ± SD	9.86 ± 4.30	8.80 ± 4.15		
Range	3–18	1–22		
**Metaphase II oocytes**			1.702	0.166
Mean ± SD	6.48 ± 3.80	5.56 ± 2.86		
Range	1–14	1–16		
**Embryo Transfer**			2.017	0.365
One embryo	6	10		
Two embryos	15	10		
Three embryos	29	30		

Comparison between Granulocyte Colony Stimulating Factor (GCSF) and Human Chorionic Gonadotropin (HCG) according to ICSI parameters

^*^The day at which HCG was injected from the beginning of the cycle

^†^The time between HCG injection day and oocytes retrieval

X2 refers to chi-square test result

t refers to student t-test

Table 3 compares the pregnancy outcomes of the two groups. We found a significant improvement in implantation rates favoring G-CSF over HCG (*P* < 0.0001). According to chemical pregnancy, In the G-CSF group, 17 (34%) women were negative, and 33 (66%) women were positive, while, in the HCG group, 35 (70%) women were negative and 15 (30%) women were positive. According to Clinical Pregnancy, In the G-CSF group, 20 (40%) women were negative, and 30 (60%) women were positive, while, in the HCG group, 37 (74%) women were negative and 13 (26%) women were positive. These findings confirm that G-CSF is significantly superior to HCG regarding implantation rate (*P* < 0.0001), chemical pregnancy (*P* = 0.0003), and clinical pregnancy (*P* = 0.0006), (Table 3).

**Table 3:** Comparison between Granulocyte Colony Stimulating Factor (GCSF) and Human Chorionic Gonadotropin (HCG) according to outcomes

Parameters	GCSF group (*n* = 50)	HCG group (*n* = 50)	t/X2	*P*-value
**Implantation rate (Sac)**			15.167#	0.0002*
0	20 (40%)	35 (70%)		
1	4 (8%)	7 (14%)		
2	23 (46%)	8 (16%)		
3	3 (6%)	0 (%)		
**Implantation rate (Pulsation)**			15.439#	0.0014*
0	20 (40%)	37 (74%)		
1	4 (8%)	5 (10%)		
2	23 (46%)	8 (16%)		
3	3 (6%)	0 (%)		
**Chemical Pregnancy**			12.981#	0.0003*
Negative	17 (34%)	35 (70%)		
Positive	33 (66%)	15 (30%)		
**Clinical Pregnancy**			11.791#	0.0006*
Negative	20 (40%)	37 (74%)		
Positive	30 (60%)	13 (26%)		

Comparison between Granulocyte Colony Stimulating Factor (GCSF) and Human Chorionic Gonadotropin (HCG) according to ICSI parameters

^*^The day at which HCG was injected from the beginning of the cycle

^†^The time between HCG injection day and oocytes retrieval

X2 refers to chi-square test result

t refers to student t-test

## Discussion

Our randomized control trial compared the efficacy of G-CSF and HCG as effective treatments in women who have undergone ICSI with a history of RIF, we found a significant improvement in pregnancy outcomes favoring G-CSF over HCG in implantation rate, chemical pregnancy, and clinical pregnancy.

RETRACTED

Scarpellini and Sbracia were the first to consider using G-CSF in reproductive medicine to treat couples who had recurrent miscarriages. The authors found that by the sixth day after ovulation, subcutaneous G-CSF injection dramatically increased live births rates (82.8%) in comparison to the control group (48.5%) (OR: 5.1, 95% CI 1.5–18.4, *P* = 0.0061) [18].

G-CSF can be given as a subcutaneous injection (SC) or intrauterine infusion (IU). The impact of G-CSF injection whether by SC or IU routes on successful implantation is still unclear. Zeyneloglu et al. compared the combined SC and IU administration of G-CSF with the only SC administration and no G-CSF administration [19]. The clinical pregnancy rates were significantly the highest with combined routes administration (64.1%), then (52.6%) with the SC route, and the least (23.5%) with no G-CSF administration, *P* = 0.0011 [19]. Also, it was the same with the live birth rates which were significantly the highest with combined SC and IU G-CSF administration (61.5%), then only SC G-CSF administration (34.2%), and the least with no G-CSF administration (23.5%), *P* = 0.001 [19].

Furthermore, more randomized clinical trials involving G-CSF administration in women with a history of miscarriage found an increased birth rate and decreased incidence of miscarriage risk [18, 20]. In addition, another study showed that it improved the thickness of the endometrium in women with a history of IVF failure [21]. This could be explained by the role of G-CSF in increasing the number of both regulatory T cells and dendritic cells which increased the expression of implantation responsible genes [7].

HCG is considered a primary signal which modulates the communication between the embryo and endometrium, improves endometrial receptivity, and triggers a gene expression cascade that leads to implantation [22, 23]. It is used whether purified or recombinant in the treatment of infertility such as with IVF treatment to help in the maturation of oocytes or with simple procedures to enhance the follicular rupture [12].

However, the effect of HCG on immune response during implantation is still unclear. Previous studies found that it boosted proangiogenic factors within the endometrium, modified uNK production, elevated Tregs, and increased trophoblastic invasion [24–26]. Mansour et al. were the first to investigate the use of IU HCG in women who underwent IVF in 2011 and found that it increased both pregnancy and implantation success rates [27].

Furthermore, Liu et al. discovered that the effect of IU HCG injections in women with RIF was different according to the stage of embryo transfer as the pregnancy rates were higher in blastocyst transplantations compared to cleaved stage embryo transfer [28]. This could be explained as women with transferred blastocyst had significantly lower ages compared to women with cleavage stage transfer [28].

RETRACTED

### Implementation of the results

Our study supported G-CSF administration over HCG to improve pregnancy outcomes in women with RIF. Unfortunately, no studies compared both treatment options. Therefore, our study added a great impact to the evidence to choose the best option to increase pregnancy outcomes in women with RIF. Only a systematic review and meta-analysis investigated different treatment options in women with RIF including HCG and G-CSF and determined the level of evidence for each treatment option in pregnancy outcomes; however, the study lacked direct comparisons between treatment options [29]. They found that G-CSF together with intrauterine peripheral blood mononuclear cells had the most promising outcomes as evidence quality for them was moderate compared to other treatment options including HCG in which the evidence quality was low or very low which was in line with our results [29].

### Limitations

In cases with RIF, treatment with G-CSF and HCG is a novel proposal for immune therapy. Few studies have been carried out to date, and many questions remain unanswered. Which patients will gain the most benefit from the treatment? What are the recommended starting dose and cycle period for treatment? What is the most effective administration route (intrauterine or systemic)? For finding answers to these problems, well-designed clinical studies with bigger sample sizes and younger women should be done.

## Conclusion

For the first time, our randomized control trial compared the efficacy of G-CSF and HCG administration on the day of embryo transfer as effective treatments in women who underwent ICSI with a history of RIF. We found a significant improvement favoring G-CSF over HCG in pregnancy outcomes such as implantation rate, chemical pregnancy, and clinical pregnancy.

Immunological therapies are of particular interest to reproductive medicine professionals. Understanding the immunological pathways of embryo implantation may open the way for developing new immunotherapies that improve pregnancy outcomes and implantation rates. Despite the small number of available studies, the results are promising.

## Data Availability

The datasets used and/or analyzed during the current study are not publically available due to the confidentiality of participants' data and the difficulty of organizing the raw data to be suitable for publication; however, they are available from the corresponding author on reasonable request.

RETRACTED

## Abbreviations

RIF: Repeated implantation failure
IVF: Several In vitro fertilization
G-CSF: Granulocyte colony-stimulating factor
HCG: Human Chorionic Gonadotropin
ICSI: Intracytoplasmic Sperm Injection
ART: Assisted reproductive technology
Tregs: Regulatory T cells
AFC: Antral follicle count
FSH: Follicle Stimulating Hormone
LH: Luteinizing Hormone
E2: Estradiol
TSH: Thyroid Stimulating hormone
AMH: Anti-Müllerian Hormone
SD: Standard deviation
SC: Subcutaneous injection
IU: Intrauterine infusion
